The article "Successful Resection of Small Intestinal Stenosis After Treatment With an Immune Checkpoint Inhibitor for Metastatic Lung Cancer in the Small Intestine: A Case Report" was published in 2024. Journal: Cureus.

# Successful Resection of Small Intestinal Stenosis After Treatment With an Immune Checkpoint Inhibitor for Metastatic Lung Cancer in the Small Intestine: A Case Report

**DOI:** 10.7759/cureus.75909

**Published:** 2024-12-17

**Authors:** Ayako Shimada, Shinnosuke Ohnaka, Masanao Nakashima, Atsushi Nagai

**Affiliations:** 1 Department of Respiratory Medicine, Shin-Yurigaoka General Hospital, Kanagawa, JPN

**Keywords:** gastrointestinal metastasis, immune checkpoint inhibitors, lung cancer, pembrolizumab, small intestinal stenosis

## Abstract

Gastrointestinal (GI) metastases from lung cancer are relatively rare, and their management strategies and outcomes in the era of immune checkpoint inhibitors are unknown. A 59-year-old man with lung cancer was hospitalized. He presented with vomiting due to a small intestinal metastasis. The metastatic lesion reduced in size with pembrolizumab treatment. However, the patient could not feed orally and required continuous central venous nutrition. Following the recurrence of a catheter-related bloodstream infection, the patient underwent small intestinal resection and gastrojejunal bypass surgery. Surgical specimens from the site of intestinal stenosis showed tumor disappearance and inflammatory cell invasion. GI stenosis due to lung cancer metastasis can persist even after effective treatment with immune checkpoint inhibitors. Therefore, surgery for GI metastases should be considered as necessary.

## Introduction

Gastrointestinal (GI) metastasis from lung cancer is relatively rare [1]. The common symptoms of GI metastasis are rupture, obstruction, and bleeding. However, many cases are asymptomatic. Emergency surgery is performed in cases of acute abdomen or severe symptoms; however, the prognosis for patients after surgery is usually poor [2].

Recently, immune checkpoint inhibitors (ICI) have been used to treat lung cancer. ICI treatment has extended the survival of some patients with advanced lung cancer. Nevertheless, outcomes and management strategies for patients with metastatic GI lung cancer treated with ICI remain unknown.

In this case report, we described a rare case of lung cancer metastasis to the intestine, in which intestinal stenosis persisted after effective ICI treatment.

## Case presentation

A 59-year-old Japanese man presented to our hospital complaining of chest pain. The patient had no comorbidities. He had a smoking history of 80 pack years. Chest computed tomography (CT) revealed an enlarged mediastinal lymph node adjacent to the tumor in the left apex of the lung, with infiltration of the thoracic vertebrae (Figure 1A). Abdominal CT revealed a small intestinal tumor (Figure 1B), which was suspected to be malignant on positron emission tomography (PET) (Figure 2).

The article "Successful Resection of Small Intestinal Stenosis After Treatment With an Immune Checkpoint Inhibitor for Metastatic Lung Cancer in the Small Intestine: A Case Report" was published in 2024. Journal: Cureus.

**Figure 1:** Contrast-enhanced CT findings of chest and abdomen. CT at diagnosis showed a metastatic tumor in the mediastinal lymph nodes (arrowhead) (A) and small intestine (arrow) (B). CT at readmission for gastrointestinal symptoms showed shrinkage of the mediastinal tumor (C) and marked enlargement of the small intestinal tumor (D). Improvement of both mediastinal and intestinal tumors was observed nine months after pembrolizumab treatment (E, F). CT, computed tomography

**Figure 2:** PET findings of chest and abdomen The PET scan showed intense FDG uptake in the mediastinal tumor (arrowhead) and in the small intestinal tumor (arrow). FDG, fluorodeoxyglucose; PET, positron emission tomography

The patient underwent bronchoscopy and from the endobronchial ultrasound-guided transbronchial needle aspiration (EBUS-TBNA) specimen of the mediastinal tumor, he was diagnosed with non-small cell lung cancer (NSCLC). His tumor had no driver mutations and a high tumor proportion score (TPS) for programmed death ligand-1 (PD-L1) (≧50%). At the time of diagnosis, it was difficult to determine whether the patient had small intestinal metastases or a primary tumor in the small intestine. Therefore, the patient was treated with chemoradiation therapy (CRT) (cisplatin+tegafur/gimeracil/oteracil and a total of 60 Gy of radiation). Following treatment, the thoracic tumor size decreased. Treatment was discontinued at the patient’s request.

Four months after the CRT, the patient presented to the emergency department with vomiting. Chest and abdominal CT revealed shrinkage of the chest tumor (Figure 1C) and enlargement of the intestinal tumor (Figure 1D). The patient’s vomiting symptoms improved after endoscopic drainage and decompression, but oral intake remained challenging. As his general condition stabilized, pembrolizumab was administered on day 7. After seven days of chemotherapy, the patient experienced vomiting and dehydration. A nasogastric tube was used for intragastric decompression. Abdominal CT revealed enlargement of the small intestinal tumor. A central venous (CV) port was implanted for nutrition, and percutaneous endoscopic gastrostomy (PEG) was performed for gastric drainage. The nasogastric tube was removed. As his general condition gradually improved and CT follow-up showed slight shrinkage of the intestinal tumor, a second dose of pembrolizumab was given on day 49 and he was discharged. Pembrolizumab was continued for six cycles.

Five months after inserting the CV port, the patient was admitted to the hospital with a fever due to a catheter-related bloodstream infection (CRBSI). Antibiotic treatment was effective. However, because of CRBSI recurrence, surgery was performed to remove the CV port. The CT scan showed a remarkable reduction in the chest and abdominal tumors (Figures 1E, 1F). As the patient was still unable to feed orally, small intestine resection and a gastrojejunal bypass were performed. The surgical specimens showed intestinal stenosis but no obvious tumor in the duodenum, both macroscopically (Figure 3A) and microscopically (Figure 3B). Microscopic findings revealed a chronic inflammatory cell infiltrate consisting mainly of lymphocytes and macrophages at the site of stenosis (Figure 3B).

The article "Successful Resection of Small Intestinal Stenosis After Treatment With an Immune Checkpoint Inhibitor for Metastatic Lung Cancer in the Small Intestine: A Case Report" was published in 2024. Journal: Cureus.

**Figure 3:** Pathology of the surgical specimen of the stenotic site of the small intestine Macroscopic findings show intestinal stenosis and roughening of the serous mucosa of the small intestine but no obvious tumor (A). Microscopic findings show no cancer cells, but a chronic inflammatory cell infiltrate consisting mainly of lymphocytes and foamy macrophages in the submucosa up to the serosal surface at the site of stenosis (Hematoxylin and Eosin staining, ×100) (B).

The patient started eating after the surgery. One month after the surgery, pembrolizumab was initiated. The patient had no difficulty passing food. Eleven months post-surgery, the cancer has not recurred.

## Discussion

In this case report, we described a patient with lung cancer with small intestinal metastasis, whose intestinal stenosis persisted after successful treatment with pembrolizumab.

Pembrolizumab is a PD-1 inhibitor and a key ICI drug. ICI works by inhibiting immune regulation by cancer cells, thereby reactivating and proliferating cytotoxic T cells to induce tumor infiltration and regression [3]. Due to the transient immune cell infiltrate, ICI can cause a phenomenon known as ‘pseudo-progression’, where the tumor size temporarily increases in the early stages of treatment [4]. Our patient experienced worsening of the small intestinal tumor (considered ‘pseudo-progression’) after treatment with pembrolizumab, followed by subsequent shrinkage of the intestinal tumor. This process suggested a good anti-tumor response, and it was expected that the obstruction in the small intestine would resolve. However, the symptoms of the small intestinal obstruction did not improve. It was difficult to determine how much of the tumor remained in the small intestine. Therefore, palliative radiotherapy was not performed. PET-CT follow-up after pembrolizumab treatment could possibly have predicted the disappearance of the tumor, but it is unclear if it could be done in the presence of inflammation. After surgery, it became clear that the thickening of the small intestinal wall that caused the intestinal obstruction was due to the infiltration of inflammatory cells. There are few reports of ICI-induced immune-related intestinal obstruction that are resolved with corticosteroid therapy. However, the reported cases did not involve obvious intestinal malignancy [5,6]. To our knowledge, this is the first report of intestinal stenosis persisting after the resolution of an intestinal metastatic tumor following ICI therapy.

The article "Successful Resection of Small Intestinal Stenosis After Treatment With an Immune Checkpoint Inhibitor for Metastatic Lung Cancer in the Small Intestine: A Case Report" was published in 2024. Journal: Cureus.

In our case, surgery was performed to relieve intestinal obstruction. Surgery in patients with advanced lung cancer carries a higher risk of surgical complications owing to the physical fragility of the patient and the spread of the tumor. For our patient, surgery was performed because there were no other dietary alternatives and no other metastases. Moreover, the patient enjoyed independent activities of daily living (ADL) and wanted surgery. On reflection, surgery could have been considered earlier because the ICI treatment was effective for his cancer and the patient had been stable for several months. Surgical removal of the intestinal obstruction enabled oral intake and greatly improved the patient’s quality of life (QOL). As in our case, surgery can improve the QOL of some patients and contribute to long-term survival. Thus, timely surgery for GI metastases should be considered on a case-by-case basis.

## Conclusions

Here, we described a patient with lung cancer metastasis to the small intestine, whose intestinal stenosis persisted after pembrolizumab treatment. Surgical resection of the small intestine revealed tumor disappearance and inflammatory cell invasion at the stenotic site.

Physicians should be aware that intestinal stenosis due to lung cancer metastasis can persist after effective ICI treatment and should consider surgical resection as necessary.
